The article "Prediction and Analysis of Dynamic Changes of College Students' Ideological and Political Changes Based on Multiple Regression" was retracted in 2023. Reasons: unreliable results or conclusions; concerns about the data; concerns about the peer review; concerns about the citations.

# Prediction and Analysis of Dynamic Changes of College Students' Ideological and Political Changes Based on Multiple Regression

**DOI:** 10.1155/2022/5323699

**Published:** 2022-07-30

**Authors:** Minhong Wang

**Affiliations:** College of Marxism, Chongqing Industry Polytechnic College, Chong Qing 401120, China

## Abstract

The construction of a harmonious society requires college students to coordinate their ideological, political, and moral qualities with social development and the needs of the times. Through the investigation and analysis of the ideological, political, and moral qualities of college students, on the one hand, we can see that the ideological, political, and moral qualities of college students are generally positive and healthy. On the other hand, it also exposes the outstanding problems in the ideological and political aspects of college students and the shortcomings of the ideological and political work in colleges and universities. This paper analyzes the dynamic changes of college students' ideological and political changes and further studies the relationship between various indicators and students' ideological and moral qualities through multiple linear regression analysis.

## 1. Introduction

Colleges and universities are an important stage for ideological and political education for young students, and the ideological and political quality of college students is also a major criterion for evaluating the effectiveness of college education. With the continuous improvement of the socialist market economic system, the rapid development of the economy, society and science, and culture, and the integration of Chinese and foreign cultures, many new changes have taken place in the ideological values of current members of society, and some even have contradictions. As the successors and builders of the cause of socialism with Chinese characteristics, the ideological and moral conditions of contemporary college students have also appeared some new changes, new characteristics, and new conditions. In some college students, there are situations such as loss of ideals and beliefs, lack of social responsibility, a weakened spirit of hard work, and a weak concept of teamwork. At the same time, due to the continuous expansion of colleges and universities in my country in recent years and the influence of the global economic recession, new requirements have also been put forward for the ideological and political education work in colleges and universities. In this environment, it is very important and urgent to further strengthen the ideological and political education work of college students. For any society, college students are the most valuable human resources and the hope and future of a country and nation. Do a good job in the ideological and political education of college students, improve their ideological and political level, and train them to be builders and successors of the socialist cause with firm political beliefs and lofty political ideals. This will ensure the healthy and sustainable development of the socialist cause with Chinese characteristics. It has long-term and important strategic significance [1, 2]. The university stage is the last stage for a person to move from school to society, and it is also an important period for the formation of young people's values, outlook on life, and moral outlook. If there is a lack of correct theoretical guidance and education in such a period, it is bound to have a negative impact [3, 4]. General Secretary Hu Jintao pointed out “College education must adhere to people-oriented, take the all-round development of college students as the goal, and guide the majority of students to learn not only to do things but also to learn to be people.”

In recent years, with the continuous development of my country's reform and opening up and the gradual improvement of the market economy system, many new situations, new characteristics, and new changes have emerged in the ideological and political quality of contemporary college students [5, 6]. On the one hand, college students' self-improvement and self-reliance, innovation and development awareness, and patriotism awareness have been significantly strengthened; at the same time, some college students also have problems such as loss of ideals and beliefs, lack of social responsibility, the weakened spirit of hard work, and teamwork concept. Under this circumstance, the task of actively promoting the ideological and political education of college students is very urgent and important.

All in all, the ideological and political quality of college students is related to the future and destiny of the country and the nation. Whether they can cultivate qualified and excellent builders and successors who meet the requirements of the cause of socialism with Chinese characteristics, it can be said that the ideological and political work of colleges and universities plays a vital role in it. [7]. Under the background of the new era, ideological and political education in colleges and universities should closely grasp the new changes in the development of the situation, start from multiple angles and levels, and actively promote and improve the ideological and political education of college students. At present, the most commonly used prediction methods are regression analysis method and decision tree method. Multiple regression analysis is one of the scientific prediction methods, and this paper will apply this method to establish multiple regression models [8–10].

## 2. Related Work

Stepwise regression: the basic idea of the stepwise regression analysis method is to automatically select the most important variables from a large number of available variables and establish a prediction or interpretation model for regression analysis. The basic idea is that the independent variables are introduced one by one, and the condition of the introduction is that the partial regression sum of squares is significant after testing. At the same time, each time a new independent variable is introduced, the old independent variables should be tested one by one, and the independent variables with insignificant partial regression sum of squares should be eliminated. In this way, it has been introduced and eliminated until neither new variables are introduced nor old variables are deleted. Its essence is to establish the “optimal” multiple linear regression equation. According to the above idea, stepwise regression can be used to screen and eliminate variables that cause multicollinearity. The specific steps are as follows: first is to perform a simple regression on each explanatory variable considered with the explanatory variable and then use the explanation that contributes the most to the explanatory variable. Based on the regression equation corresponding to the variable, the remaining explanatory variables are gradually introduced. After a stepwise regression, the explanatory variables that remained in the model were both significant and did not have severe multicollinearity.

### 2.1. MATLAB

MATLAB is commercial mathematical software produced by MathWorks in the United States. It is used in data analysis, wireless communication, deep learning, image processing and computer vision, signal processing, quantitative finance and risk management, robotics, control systems, and other fields. MATLAB is a combination of the words matrix and laboratory, which means matrix factory (matrix laboratory). The software mainly faces the high-tech computing environment of scientific computing, visualization, and interactive programming. It integrates many powerful functions such as numerical analysis, matrix calculation, scientific data visualization, and modeling and simulation of nonlinear dynamic systems in an easy-to-use window environment for scientific research, engineering design, and many sciences that must perform the effective numerical calculation. Realm provides a comprehensive solution and is largely free from the editing mode of traditional noninteractive programming languages [11, 12] (e.g., C, Fortran). MATLAB, Mathematica, and Maple are known as the three major mathematical software. It is second to none in numerical computing among mathematical technology applications. As the same time, we use the Row matrix operations, plotting functions, and data implementing algorithms, creating user interfaces, interfacing programs in other programming languages, etc. The basic data unit of MATLAB is a matrix, and its instruction expression is very similar to the form commonly used in mathematics and engineering. Therefore, it is much simpler to use MATLAB to solve problems than to use C, FORTRAN, and other languages to complete the same thing, and MATLAB also absorbs the advantages of software such as Maple, making MATLAB as powerful mathematical software. Also we added support for C, FORTRAN, C + +, and JAVA in the new version. MATLAB is a collection containing a large number of computational algorithms. It has more than 600 mathematical operation functions used in projects, which can easily realize various calculation functions required by users. The algorithms used in the function are the latest research results in scientific research and engineering computing and have undergone various optimizations and fault tolerance processing [13]. In general, it can be used in place of low-level programming languages such as C and C++. With the same computational requirements, the programming effort using MATLAB is greatly reduced. These functions of MATLAB range from the simplest and most basic functions to complex functions such as matrices, eigenvectors, and fast Fourier transforms. The problems that functions can solve generally include matrix operations and the solution of linear equations, differential equations and partial differential equations, symbolic operations, Fourier transform and statistical analysis of data, optimization problems in engineering, sparse matrix operations, Various operations on complex numbers, trigonometric functions and other elementary mathematical operations, multidimensional array operations, and modeling dynamic simulations. In the development environment, it makes it easier for users to control multiple files and graphics windows; in terms of programming, it supports function nesting and conditional interruption; in terms of graphics, there are more powerful graphics annotation and processing functions, including, in terms of input and output, you can directly connect to Excel and HDF5[14].

## 3. Our Model

### 3.1. Analysis of the Significant Influencing Factors of College Students' Ideological and Political Changes

The personal socialization environment of college students is a direct factor affecting the ideological and political education of college students [15]. It mainly includes two aspects, one is the “social setting”, that is, social institutions closely related to college students, mainly including families, schools, television, books, newspapers, the Internet, and radio; other social subjects other than college students who have a close relationship with life and study mainly include parents, lovers, relatives of the same age, friends or classmates, class teachers or counselors, and classroom teachers. During the implementation of the survey, various main factors included in the above-mentioned “social settings” and “social subjects” were measured in college students' “morality and ethics”, “ideal beliefs”, “love and marriage”, “handling affairs”, “talent employment”, “interpersonal communication”, “hobbies”, “entertainment consumption,” and “leisure life”. Tables 1 and 2 show the main results of the survey [16].

#### 3.1.1. Parents and Families Are Extremely Important Influencing Factors of College Students' Values, Morality, and Ethics

A person's life is inseparable from the family, and the family and its parents play a very important role in the growth of young people. The data in Table 1 show that among the “social setting” factors that affect the ideological and political status of college students, the influence of family on college students' “morality and ethics”, “ideal beliefs”, “love and marriage”, and “handling of affairs” is all in the First, the proportions are 45.2%, 28.5%, 37.4%, and 44.6%, respectively [6]. It is also in second place in “successful employment” (19.3%) and “interpersonal communication” (30.7%). For college students who have left their families to study abroad, family and parents are still the main factors affecting their ideological and political status. The results in Table 2 also show that college students are most willing to listen to their parents' opinions in terms of “morality and ethics,” “handling affairs,” “love and marriage,” and “successful employment.” The proportions are 52.2%, 47.2%, and 33.7%, and 27.2%, respectively; in terms of “ideal beliefs” (24.9%) and “interpersonal communication” (34.9%), the importance of parents' opinions also ranks second. These phenomena fully demonstrate the position and weight of parents in the minds of college students. When making decisions about life events, they first consider the opinions of their parents. It is worth noting that the “ideal beliefs” of college students are affected by many factors, and the proportion of choosing “other people” occupies the first place with 27.5% [17]. This shows that the factors affecting college students' “ideological beliefs” are diverse. Except for parents, friends, and classmates, the factors affecting college students are not the same [18].

#### 3.1.2. School Is the Main Factor Affecting the Employment and Interpersonal Communication of College Students

From the data in Table 1, it can be seen that schools play a leading role in “interpersonal communication”, “talent employment”, and “hobbies”, accounting for 49.3%, 35.7%, and 20.6%, respectively. It has the second-largest influence on “dealing with affairs” (30.1%) and “leisure life” (19.4%); in “ideals and beliefs” (21.9%), “morality and ethics” (17.1%) and “love and marriage” (13.8%) play the third influential role [19]. These situations show that schools have an important influence on the development of college students' ideological and political quality. From the data in Table 2, it can be found that from the perspective of the ideological and political education workforce, counselors and class teachers are in the “successful employment” (23.8%), “handling affairs” (12.6%), and “morality and ethics” (11.6%). It also has a direct and important influence on the ideological and political quality of college students.

In addition, social practice activities as important teaching content and teaching links are not only an important influencing factor of college students' ideological and political education but also an effective carrier of college students' ideological and political education. The survey shows that “participating in public welfare social practice” is listed as the first effective way for ideological and political education by college students, accounting for 65.1%. At the same time, among the activities carried out by the Communist Youth League in colleges and universities, campus cultural activities, youth volunteer activities, community activities, “Challenge Cup” activities, and “Three Going to the Countryside” activities are the most popular among college students, with 48.4% of them being selected, and 48.4% of them being selected. 47.6%, 30.0%, 29.8%, and 29.1%. These activities belong to the category of social practice and play a positive role in promoting college students to contact the society, understand society, and enhance their hands-on ability. However, the lack of social practice bases and positions makes it difficult to meet the needs of most students. The survey shows that 66.1% of college students have not engaged in on-campus work-study work, and 40.8% have not engaged in any economic activities. Among the economic activities they have engaged in, tutoring (37.2%) and part-time work (29.7%) are their main social practices. It can be seen from this that contemporary college students have few opportunities for social practice in ideological and political education, and their social practice ability has not been effectively improved, which leads them to place great expectations on social practice. At the same time, most colleges and universities believe that there are problems in the base construction, time arrangement, funding guarantee, and system establishment of social practice. Therefore, it is necessary to pay more attention to and strengthen the social practice work of college students, strive for local support, strengthen the construction of social practice bases, and guide students' social practice activities to develop in a long-term, positional, project-based, and hierarchical direction. Efforts should be made to explore the daily form of social practice activities and use weekends or other spare time to choose the community near the school as a fixed social practice base to carry out social practice activities.

#### 3.1.3. Peer Groups Play an Important Role in College Students' Hobbies and Daily Behaviors

The peer groups of college students mainly include classmates, roommates, and members of clubs. Because college students get along with their peers day and night, have the same hobbies, similar life experiences, and have the same troubles and needs, they influence each other infrequent interactions, and especially in specific behaviors, they play a dominant role. The survey data in Table 2 show that in terms of “entertainment consumption” (56.6%), “leisure life” (55.3%), “hobbies” (55.2%), and “interpersonal communication” (43.2%), their influences are all listed No. 1. The influence of “handling affairs” (20.9%) ranks second, and the influence of “ideal and belief” (22.2%), “love and marriage” (19.5%), and “talent employment” (15.0%) and the other three influence of each aspect ranks third. It can be seen that peer group plays a very important role in the life and study of college students.

The influence of peer groups is mainly through good friends. The survey shows that middle school classmates (85.1%), college classmates (76.0%), and roommates (73.5%) are the main objects within the scope of college students' good friends. At the same time, the good friends of college students have also included some new objects, such as fellow villagers (32.7%), members of group organizations or student unions (17.6%), members of clubs (15.0%), netizens (11.7%), class teachers (9.8%), classroom teachers (9.8%), and counselors (9.1%). Once you understand the main scope of good friends for college students, you can start with these objects in a targeted manner and achieve the goal of ideological and political education through the familiarity and example of good friends. At the same time, the dormitory atmosphere is also an important factor affecting the ideological and political education of college students. According to the survey, “study” (51.3%) is the eternal theme discussed by college students in the dormitory. “Daily trifles” (32.3%), “employment prospects” (31.7%), “current affairs news” (31.3%), and “things happening in the class and school” (29.3%) were also discussed in the “squatting meeting” main content (see Table 3). Therefore, in a certain sense, ideological and political education is not only preaching political theory but also achieves its goal through comprehensive interpersonal interaction.

### 3.2. Multiple Regression Analysis

Stepwise regression is a common mathematical method for selecting regressors in multiple linear regression models [5, 10]. The basic idea is, according to the size of the effect of factors *x*_1_, *x*_2_, ..., *x*_*m*_ on *y*, the factors are introduced into the regression equation one by one from large to small. For the factors that have been introduced into the equation, after the introduction of new factors, they may be eliminated from the equation at any time because they have no significant effect on *y*. After the variable is introduced, it can also be put back in order to obtain a regression equation with some optimal properties [12] and study the regression between a dependent variable and two or more independent variables. Also known as multiple linear regression, it reflects the law that the number of a phenomenon or thing changes correspondingly with the change of the number of a variety of phenomena or things. We have used a statistical method for establishing the quantitative relations of linear or nonlinear mathematical models among multiple variables. In regression analysis, if there are two or more independent variables, it is called multiple regressions. In fact, a phenomenon is often associated with multiple factors. It is more effective and practical to predict or estimate dependent variables by the optimal combination of multiple independent variables than to predict or estimate only one independent variable. Therefore, multivariate linear regression is more practical than univariate linear regression. When all the variables introduced into the equation have reached a significant level, and at the same time, no new variables can be introduced, the stepwise regression is announced, and the optimal equation obtained at this time is between the least independent variables and the best fitting effect. The optimal equilibrium is reached [20]. It should be pointed out that the reason why it is emphasized here that the independent variables included in the regression equation should be as few as possible without affecting the fitting effect of the regression equation is that the more independent variables, the higher the requirements for data sources [21]. Many variables must be measured during prediction, which undoubtedly increases the difficulty of implementation. The effect of prediction will also decline with the inaccuracy of some variables, thereby increasing the instability of the system [12]. The following is a stepwise regression analysis of the above 16 variables that significantly affect the duration of events to determine the best combination of variables for predicting the dynamic changes in college students' ideological and political changes and establish a multiple linear regression model. In this study, the stepwise regression function [22] in the MATLAB statistical toolbox is used to select variables for the multiple regression equation, and the optimal variable combination is shown in Figure 1. The graph shows the regression coefficients and confidence intervals for each variable, and the terms shown in white (confidence intervals are indicated by solid lines) are variables that have been selected for the model; confidence intervals shown in grey are indicated by dashed lines of terms are variables that are not in the model. Building a harmonious society requires college students to coordinate their ideological, political, and moral qualities with social development and the needs of the times. Through the investigation and analysis of college students' ideological and political moral qualities, on the one hand, we can see that college students' ideological and political moral quality is positive, healthy, and upward on the whole; on the other hand, it also exposes the outstanding problems in college students' ideological and political work and the deficiencies in college students' ideological and political work.

The parameters of the regression equation are shown in Figure 2. The figure shows the regression coefficient and confidence interval of each variable, the root mean square of the current model error, the amount of the corresponding variable explained by the model, the statistic *F* of the regression model, and the significant probability *P* associated with the analysis.

The 16 variables in Figures 1 and 2 are interpersonal communication, talent and employment, handling affairs, morality, participation in public welfare social practice, laws and regulations, love and marriage, talent and employment, ideals and beliefs, social responsibility, school uniforms, and friends' influence, teacher teaching, parental requirements, self-discipline, and moral restraint. As can be seen from Figure 1, after step-by-step regression analysis, variables 2 to 9, namely career and employment (*x*_1_), handling affairs (*x*_2_), morality and ethics (*x*_3_), participation in public welfare social practice (*x*_4_), laws and regulations (*x*_5_), love marriage (*x*_6_), successful employment (*x*_7_), and ideal beliefs (*x*_8_), were selected into the regression equation, while other variables were eliminated from the original regression equation. Using *y* to represent the event duration, the established multiple linear regression model is

(1) $$\begin{array}{c} y=9.3x_{1}+19.4x_{2}+5.1x_{3}+8.4x_{4}+5.5x_{5}+26.4x_{6}+4.5x_{7}+58.7x_{8}+28.9. \end{array}$$

It can be seen from the above formula that among the eight independent variables of the equation, ideal beliefs have the greatest impact on ideological and political changes. In addition, two variables, dealing with affairs and love and marriage, also have a large effect on the duration.

The constant term in the regression equation is large, which makes the equation predict ideological and political changes, even if the values of all variables are 1, the minimum predicted value is 28.9. That is to say, for small events with small changes, the prediction of the equation will generally be too large.

As can be seen from Figure 2, the optimal regression equation obtained by stepwise regression is significant (*P*  = 0).

## 4. Multiple Regression Model Effect Test

In order to examine the validity of the regression model, 170 groups of actual event data are used to test the prediction effect of the regression equation. The results are shown in Figure 3.

Figure 3 shows that the predicted value of most events is still relatively close to the actual value. The correlation analysis shows that the predicted value has a good correlation with the actual value, and the correlation coefficient is 0.8573. The results predicted by the multiple linear regression model can basically reflect the real dynamic changes. In order to illustrate the prediction effect of the regression model more clearly and intuitively, the difference between the predicted value and the actual value is counted below, and the statistical result is given in a histogram, as shown in Figure 4.

As can be seen from Figure 4, among the 170 test samples, 1 has a prediction error of 0, 59 are between 0 and 10, 59 are between 10 and 20, and 59 are between 20 and 30. There are, 21 more than 30. That is to say, about 35% of ideological and political changes have a prediction error of less than 10, and 70% of events have a prediction error of less than 20.

In order to verify the significance of the prediction of the developed multiple regression model, this study took the significance level *α*=0.0 and performed a nonparametric one-way ANOVA. The results show that  *P*=0.0058 < *α*, which shows that the multiple linear regression equation has significant statistical significance, and the prediction can basically obtain a satisfactory prediction effect. Finally, we use the above data to prove the feasibility of our model.

## 5. Conclusion

This paper conducts a step-by-step regression analysis of the ideological and political change group data of 660 students in a university and establishes the ideological and political dynamics with 8 variables of handling affairs, morality, participation in public welfare social practice, laws and regulations, love and marriage, successful employment, and ideals and beliefs. The multiple linear regression model of change prediction was used, and the prediction accuracy of the prediction model was tested with another 170 sets of data. The correlation coefficient between the predicted value and the actual value was as high as 0.8573. This shows that the multiple linear regression model proposed in this paper can more realistically reflect the duration characteristics of events and can basically obtain satisfactory prediction results. If more and more detailed data can be obtained for the establishment of multiple regression prediction models, it is believed that the prediction accuracy will be further improved. However, due to the extensiveness, randomness, and complexity of the factors that affect the duration of events, the author believes that even the best algorithms cannot predict the duration of events very accurately. It is hoped that the research in this paper can provide some guidance and reference for the development of college students' ideological and political development.

## Figures and Tables

**Figure 1:** Stepwise regression diagram.

**Figure 2:** Stepwise regression diagnosis table.

**Figure 3:** Comparison of predicted and actual values of multiple regression equations.

**Figure 4:** Statistical chart of test error.

**Table 1:** The influence of different social settings on the ideological and political education of college students.

	The first institution	The second body	The third agency
Moral and ethical	Family (45.2%)	Books, newspapers, and magazines (21.5%)	School (17.1%)
The ideal faith	Family (28.5%)	Books, newspapers, and magazines (28.4%)	School (21.9%)
Love marriage	Family (37.4%)	Others (26.6%)	School (13.8%)
Handle affairs	Family (44.6%)	School (30.1%)	Books, newspapers, and magazines (10.0%)
Up employment	School (35.7%)	Family (19.3%)	Books, newspapers, and magazines (16.6%)
Interpersonal communication	School (35.7%)	Family (30.7%)	Books, newspapers, and magazines (7.6%)
Interests and hobbies	School (49.3%)	Books, newspapers, and magazines (19.8%)	TV (16.5%)
Entertainment consumption	TV (23.9%)	Internet (15.9%)	School (15.9%)
Leisure life	Internet (21.8%)	School (19.4%)	TV (17.9%)

**Table 2:** The degree of influence of different social subjects on the ideological and political education of college students.

	The first object	The second object	The third object
Moral and ethical	Parents (52.2%)	Others (13.4%)	Class teacher or counselor (11.6%)
The ideal faith	Others (27.5%)	Parents (24.9%)	Friends or classmate (22.2%)
Love marriage	Parents (33.7%)	Others (23.1%)	Friends or classmate (19.5%)
Handle affairs	Parents (47.2%)	Friends or classmate (20.9%)	Class teacher or counselor (12.6%)
Up employment	Parents (27.2%)	Class teacher or counselor (23.8%)	Friends or classmate (15.0%)
Interpersonal communication	Friends or classmate (43.2%)	Parents (34.9%)	Others (8.1%)
Interests and hobbies	Friends or classmate (55.2%)	Others (24.0%)	Lovers (8.1%)
Entertainment consumption	Friends or classmate (56.6%)	Others (14.8%)	Parents (11.5%)
Leisure life	Friends or classmate (55.3%)	Others (15.7%)	Lovers (15.2%)

**Table 3:** The main content of communication between college students and their roommates.

Communication content	Percentage (%)
Learning	51.3
Daily chores	32.3
Employment prospects	31.7
Current news	31.3
What's going on in class and school	29.3
Men's and women's emotion	18.7
Personal mood	17.8
Television and movies	16.1
Sports news	15.4
Evaluation of the opposite sex	12.7
Consumption	12.5
Entertainment news	10.5

## Data Availability

The experimental data used to support the findings of this study are available from the corresponding author upon request.
